This article has been retracted.

# Apelin Alleviates Meniscus Endothelial Cell Apoptosis in Osteoarthritis

**DOI:** 10.1155/2022/3556372

**Published:** 2022-01-13

**Authors:** Dinggui Lu, Jihua Wei, Jian Chen, Jingjie Zhao, Jiajia Wang, Yuanxun Gong, Liuzhi Wei, Qiuju Wei, Huadeng Ban, Yueyong Li, Zechen Wang, Changtai Luo, Haidong Zhou, Jiajia Shen, Qiujiao Liao, Siyuan He, Weiyang Zhang, Qunqiang Luo, Kegong Xie, Jian Song, Lingzhang Meng

**Affiliations:** ^1^Center for Systemic Inflammation Research (CSIR), School of Preclinical Medicine, Youjiang Medical University for Nationalities, Baise, Guangxi Province, China; ^2^Department of Traumatology, The Affiliated Hospital of Youjiang Medical University for Nationalities, Baise, Guangxi Province, China; ^3^Department of Sport Medicine, The Affiliated Hospital of Youjiang Medical University for Nationalities, Baise, Guangxi Province, China; ^4^Department of Spinal Surgery, The Affiliated Hospital of Youjiang Medical University for Nationalities, Baise, Guangxi Province, China; ^5^Life Science and Clinical Research Center, The Affiliated Hospital of Youjiang Medical University for Nationalities, Guangxi Province, China; ^6^School of Pharmacy, Youjiang Medical University for Nationalities, Baise, Guangxi Province, China; ^7^Department of Foot and Hand Surgery, The Affiliated Hospital of Youjiang Medical University for Nationalities, Baise, Guangxi Province, China; ^8^Department of Interventive Medicine, The Affiliated Hospital of Youjiang Medical University for Nationalities, Baise, Guangxi Province, China

## Abstract

Osteoarthritis (OA) is a degenerative disease characterized by articular cartilage and/or chondrocyte destruction, and although it has long been considered as a primary disease, the importance of meniscus endothelial cell modulation in the subchondral microenvironment has recently drawn attention. Previous studies have shown that apelin could potentially inhibit cellular apoptosis; however, it remains unclear whether apelin could play a protective role in protecting the endothelium in the OA meniscus. In this study, with the advantages of single-cell RNA sequencing (scRNA-seq) data, in combination with flow cytometry, we identified two endothelial subclusters in the meniscus, featured by high expression of Homeobox A13 (HOXA13) and Ras Protein-Specific Guanine Nucleotide Releasing Factor 2 (RASGRF2), respectively. Compared with control patients, both subclusters decreased in absolute cell numbers and exhibited downregulated APJ endogenous ligand (APLN, coding for apelin) and upregulated apelin receptor (APLNR, coding apelin receptor). Furthermore, we confirmed that in OA, decreased endothelial cell numbers, including both subclusters, were related to intrinsic apoptosis factors: one more relevant to caspase 3 (CASP3) and the other to BH3-Interacting Domain Death agonist (BID). In vitro culturing of meniscal endothelial cells purified from patients proved that apelin could significantly inhibit apoptosis by downregulating these two factors in endothelial cell subclusters, suggesting that apelin could potentially serve as a therapeutic target for patients with OA.

## 1. Introduction

Osteoarthritis (OA), a degenerative joint disease, is generally associated with obesity and ageing. Although overexercise can elevate the risk of OA, it is usually considered a genetically driven disease [1]. In recent years, the pathological variations of the cellular components, especially the pathogenic meniscus and vasculature in OA, have garnered increasing attention [2–4]. Although the vasculature in the joint was observed to be abnormal in patients with OA [1, 5], its molecular mechanism is still difficult to understand, as research is impacted by a technique limitation in acquiring sufficient endothelial cells. The rise of the scRNA-seq technique allows for exploring transcriptome in a high-throughput manner at a single-cell level so that the endothelial cell heterogeneity can be studied more conveniently [6, 7]. Notably, endothelial cells in different organs (e.g., brain, lung, and heart) exhibit tissue-specific heterogeneity, characterized by molecular signatures such as those related to pathways and cell-surface markers [6–8]. Particularly, research on tissue-specific endothelial cell heterogeneity will help to understand the development of various diseases.

In this study, scRNA-seq data of meniscus biopsies isolated from patients with OA were adopted, and endothelial cells were isolated to explore heterogeneity by complying with genetic features. On this basis, the degenerative meniscus vasculature in endothelial cell subclusters of patients with OA was confirmed. Furthermore, intrinsic apoptosis factors (i.e., CASP3 and BID) were reported to be related to two meniscus endothelial cell subclusters in patients with OA.

Apelin is a pleiotropic peptide known as an adipokine [9]. It has been shown to possess various biological activities, such as attenuation of endoplasmic reticulum stress and apoptosis in ischemic stroke [10], influencing mitosis and apoptosis in intestinal cell lines [11], and inhibiting bone marrow mesenchymal stem cell apoptosis [11]. However, whether this molecule could protect the meniscus endothelial cells in patients with OA is still unknown. In this study, the discovery of upregulation of the apelin receptor (APLNR), a marker for endothelial cell injury [12], prompted us to investigate the role of apelin as a potential therapeutic method to alleviate meniscal endothelium injury in patients with OA.

This study reported that apelin alleviates meniscal endothelial cell apoptosis in patients with OA by inhibiting CASP3 and BID in different EC clusters.

## 2. Materials and Methods

### 2.1. Data Availability

The data and code generated or analyzed in this study are available from the corresponding author upon reasonable request.

### 2.2. Acquisition of Meniscus scRNA-seq Data

The human meniscus scRNA-seq data were provided by Sun et al. [13], retrieved from the NCBI Gene Expression Omnibus database accessed at GSE133449. The dataset consisted of three meniscus biopsies isolated from patients during supra-knee amputation but without any history of OA, rheumatoid arthritis, or other diseases related to the meniscus. Therefore, the samples were used as controls. In addition, four meniscal biopsies were isolated from patients with OA during knee arthroplasty surgery. In the present study, cells with at least 50 genes, and genes expressed in at least three cells were analyzed.

### 2.3. Human Meniscus Biopsies

Overall, control meniscus biopsies were isolated from 52 patients who underwent arthroscopic surgery after acute injury to the meniscus. A total of 84 patients with OA having undergone arthroscopic surgery provided biopsies. Each patient underwent a single biopsy. The biopsies were taken for the pathological examination. Furthermore, none of the patients had a history of knee-related disease.

### 2.4. Antibodies

In this study, the antibodies used for flow cytometry were as follows: 7-AAD (Invitrogen, #A1310), anti-human CD45 (clone HI30, eBiosciences, # 48-0459-42), anti-PECAM1 (clone WM59, Biolegend, #303106), anti-human/mouse/rat HOXA13 (Biorbyt, #orb461791), anti-human cleaved caspase 3 (clone Asp175, Cell Signalling, #9602), anti-human/mouse/rat RASGRF2-Biotin-conjugated (Biocompare, #MBS544685), anti-Bid Cleavage Site antibody (abcam, ab10640), streptavidin-APC (Invitrogen, #17-4317-82), and anti-human APJ/APLNR (BIOSS, #bs-2430R-Cy7).

### 2.5. Flow Cytometry

The meniscus biopsies were cut into small pieces and digested with collagenase IV (Gibco, #17017-019) at 37°C for 30 min. In addition, PBS/0.5%BSA/2 mM EDTA was added 10 min before the completion of digestion. The single-cell suspension was produced by filtering through a 100 *μ*m cell strainer. The nonspecific binding was blocked with an Fc receptor binding inhibitor (Invitrogen, #14-9161-73) for 15 min. Subsequently, the cells were washed with cold PBS/0.5%BSA and incubated with antibodies for 15 min on ice. The cells were fixed and permeabilized for intracellular staining with a commercial Cytofix/Cytoperm kit (BD, #554717). After washing twice with PBS/0.5%BSA, the cells were incubated with the antibodies for 20 min on ice. Specific to biotinylated anti-RASGFR2, the cells were washed twice and then incubated with streptavidin-APC for another 15 min on ice. After washing twice, the cells were resuspended in PBS/0.5%BSA/2 mM EDTA. Biopsies were measured using a flow cytometer (Thermal Fisher Attune NxT).

### 2.6. Fluorescence-Activated Cell Sorting

After the surface staining of fluorescent-labeled antibodies, the cells from patients with OA were placed into a FACS cell sorter (BD FACSMelody) to produce purified meniscus endothelial cells. The 7-AAD-CD45-PECAM1+ cells (living endothelial cells) were harvested. The produced endothelial cells with a purity ≥98% were analyzed in depth (Supplementary Figure 1).

### 2.7. Cell Culture

Human primary meniscus endothelial cells were obtained by fluorescence-activated cell sorting, as described above. After sorting, the cells were resuspended in an EC culture medium (StemCell, #08000) containing penicillin-streptomycin-neomycin (Sigma-Aldrich, #P4083) at a density of 2 × 10^4^ cells/well. Subsequently, the cells were cultured overnight in 48-well plates. After adding apelin (100 nM, Sigma-Aldrich, #A6469) and/or ML221 (blocking apelin receptor, 100 nM, Sigma-Aldrich, #SML0919) for 8 h, the cells were harvested for indepth analysis.

### 2.8. Real-Time PCR

After the meniscus endothelial cells purified from patients with OA were cultured for 24 h, mRNA was extracted using the TurboCapure mRNA kit (QIAGEN, #72251). cDNA was synthesized using TaqMan Reverse Transcription Reagents (Invitrogen, #4304134), and qPCR was performed using the Brilliant III Ultra-Fast QPCR Kit (Agilent, #60083) with a LightCycler 96 machine (ROCHE). Primers used for qPCR: APLN forward 5′-GTCTCCTCCATAGATTGGTCTGC-3′ and reverse 5′-GGAATCATCCAAACTACAGCCAG-3′; CASP3 forward 5′-GAAATTGTGGAATTGATGCGTGA-3′ and reverse 5′-CTACAACGATCCCCTCTGAAAAA-3′; BID forward 5′-ATGGACCGTAGCATCC CTCC-3′ and reverse 5′- GTAGGTGCGTAGGTTCTGGT-3′; GAPDH forward 5′-GGAGCGAGATCCCTCCAAAAT-3′ and reverse 5′-GGCTGTTGTCATACTTCTCATGG-3′ (internal control).

### 2.9. Statistical Analysis

Statistical analysis was performed using GraphPad Prism v5 software (La Jolla, USA). A nonparametric test was used for the data analysis. Results are presented as the mean ± SD in dot plots. NS: no significance (*p* > 0.05), ^∗^*p* < 0.05, ^∗∗^*p* < 0.01, ^∗∗∗^*p* < 0.001.

## 3. Results

### 3.1. Identification of Meniscus Endothelial Cells

It is reported that in meniscus, the immune cells and vasculature mainly distributed in the red zone [14]. Meniscus scRNA-seq data were analyzed using the *R* package Seurat [15], and the cells were clustered at a resolution of 0.6. Overall, nine clusters were separated from the control meniscus biopsies, while 11 clusters were separated from the OA biopsies (Figure 1(a)). To identify endothelial cells, three endothelial cell feature genes (i.e., CD93, CDH5, and PECAM1) [16, 17] were employed (Figure 1(b) and Supplementary Figure 2). In the control meniscus, cluster 6 was clearly identified as the endothelial cells for the high expression of the three feature genes observed. In OA biopsies, cluster 10 was identified as endothelial cells because of the high expression of CD93, CDH5, and PECAM1. Although, cluster 5 also exhibited the obvious expression of CD93, a high expression of monocyte/macrophage markers, CD14, and MS4A7 [13, 18] was observed (Figure 1(b) and Supplementary Figure 2). Cluster 5 was excluded from the subsequent analysis to diminish ambiguous results because it was reported that certain monocyte subsets could also express CD93 [19].

As revealed from the scRNA-seq measurements, endothelial cells comprised approximately 2% (cluster 6) of total meniscus cells in the controls, whereas they decreased to about 1% (cluster 10) in patients with OA. Flow cytometry experiments were performed to compare the meniscus endothelial cells between the controls and patients with OA to confirm these phenomena. Consistently, endothelial cells decreased by 36% in patients with OA compared with the control biopsies (Figures 1(d) and 1(e)). The decreased endothelial cells could result from facilitated apoptosis, especially in chronic inflammation [20, 21].

### 3.2. Meniscus Endothelial Cells Are Heterogeneous

Isolated endothelial cells from scRNA-seq data were integrated to compare the meniscus endothelial cells between the control and patients with OA. The unbiased subclustering analysis identified two subpopulations in the total meniscus endothelial cells (Figure 2(a)). Notably, HOXA13 was predominantly expressed in the first subcluster, whereas RASGRF2 was preferentially expressed in the second subcluster; therefore, these two subclusters were termed as EC (HOXA13) and EC (RASGRF2), respectively (Figures 2(a) and 2(b)). The genetic profiles of the two subclusters were compared (Supplementary Table 1) to confirm the heterogeneity of the meniscus endothelial cells. The heat map shows the disparity of the top 10 genes between the two subclusters (Figure 2(c)). Based on the differences in genetic profiles between the meniscus endothelial cell subclusters, the gene set enrichment analysis showed that EC (HOXA13) plays a pivotal role in the cellular response to organic substances, responding to chemical stimulus, regulation of response to stimulus, and modulation of extracellular region. In addition, another EC subcluster EC (RASGRF2) could potentially participate in the neutrophil apoptotic process and modulation of type V collagen (Figure 2(d)). To compare the above two subclusters between the controls and patients with OA, split UMAPs showed that both subclusters decreased in a number of patients with OA (Figure 2(e)). Moreover, flow cytometry analysis of isolated meniscus biopsies from patients showed decreased numbers of endothelial subclusters (Figures 2(f) and 2(g)).

### 3.3. Upregulated Intrinsic Apoptosis Factors in Meniscus Endothelial Cell Subclusters

To explore the factors potentially resulting in decreased meniscus endothelial cell numbers in patients with OA, differentially expressed genes (DEGs) were calculated from the scRNA-seq data. Overall, 2831 DEGs were identified in EC (HOXA13), and 5297 DEGs were identified in EC (RASGRF2) (Figure 3(a), Supplemental Tables 2 and 3). The most significant DEGs were labeled in volcano plots by cluster. Specifically, drastically decreased APLN was identified in both the subclusters (Figure 3(a), Supplementary Figure 3) since it was reported that apelin significantly inhibits apoptosis [9, 22–25]. Interestingly, both meniscal endothelial subclusters exhibited upregulated expression of APLNR, coding the apelin receptors (Figure 3(a), Supplementary Figure 3). Consistently, meniscus endothelial cells purified from patients showed downregulated APLN expression in patients with OA (Figure 3(b)). Moreover, flow cytometry analysis showed that APLNR was upregulated in both meniscal endothelial subclusters in patients with OA (Figures 3(c) and 3(d)), demonstrating that meniscus endothelial cells in patients with OA were severely injured and undergoing apoptosis [12]. This observation revealed that apelin could function as a therapeutic target against apoptosis in meniscal endothelial cells in both subclusters.

Apoptosis-related genes were extracted from DEGs (Supplemental Tables 2 and 3) and plotted by subclusters (Figure 3(e)) to determine the genes potentially involved in the apoptosis of meniscus endothelial cells. It is noteworthy that CASP3 showed upregulated expression in EC (HOXA13) of patients with OA, while BID was upregulated in EC (RASGRF2) of patients with OA. In addition, other apoptosis-related genes selected from DEGs (e.g., CASP7, FAS, TNFRSF1A, and TNFSF10) were downregulated in patients with OA. Notably, CASP3 and BID could function as intrinsic apoptosis genes [26–28], while FAS, TNFRSF1A, and TNFSF10 are extrinsic apoptosis genes [29]. This observation suggests that decreased meniscus endothelial cell numbers in patients with OA could be attributed to intrinsic apoptosis rather than extrinsic apoptosis.

### 3.4. Apelin Alleviates Meniscus Endothelial Cell Apoptosis

Fluorescent-activated cell sorting experiments were performed to acquire highly purified endothelial cells from meniscus biopsies to verify whether apelin can inhibit intrinsic apoptosis in the meniscus endothelial cells of patients with OA. The isolated endothelial cells were treated with BSA, APLN, or APLN and its receptor blocker (ML221) for 8 h. As indicated by flow cytometry analysis, early apoptosis (annexin V + PI-cells) of meniscus endothelial cells isolated from patients with OA was significantly inhibited by apelin, whereas it was abolished by ML221, a blocker of the apelin receptor [30] (Figures 4(a) and 4(b)). To clarify whether it could be attributed to apelin's effect on intrinsic apoptosis genes, RNA was extracted from cultured meniscus endothelial cells isolated from patients with OA. As indicated by the quantitative PCR analysis, CASP3 and BID expression levels were inhibited by apelin treatment and restored by blocking the apelin receptor (treated with ML221). Furthermore, flow cytometry was performed to analyze cleaved caspase 3 (activated caspase 3) in EC (HOXA13) and cleavage site Bid in EC (RASGRF2). Consistently, apelin significantly inhibited these two activated intrinsic apoptosis factors in endothelial subclusters, and treatment with ML221 restored their expression.

## 4. Discussion

Blood vessels modulate the tissue microenvironment and provide nutrients and immune factors affecting other cells [3, 31], in which endothelial cells play a significant role in maintaining tissue homeostasis and in the development of various diseases. Therefore, extensive studies have been conducted to explore the biological and pathological features of endothelial cells in the brain, lung, heart, skin, and other tissues [6–8, 12]. Existing studies indicate that tissue-specific endothelial cells exhibit distinguished subclusters, genetic profiles, and biomarkers among diseases. However, biological/pathological features of meniscus endothelial cells have rarely been studied due to extremely poor vascularity in the human meniscus [32], resulting in meniscus endothelial cell heterogeneity still considered an enigma. Accordingly, it is more urgent to illustrate the molecular mechanisms of meniscus endothelial cells under pathological conditions (e.g., in OA).

This study used data from scRNA-seq of meniscal biopsies isolated from patients with OA [16]. This method effectively maintained cellularity, especially for rare cells, including endothelial cells, and allowed exploring the transcriptome of meniscus endothelial cells in a high-throughput manner. Indeed, clarifying the genetic features of meniscus endothelial cells will help gain insights into the development of OA [33] and cultivate new strategies against this disease. Normally, two feature genes were adopted to identify specific cell types; however, in this study, three feature genes (CD93, CDH5, and PECAM1) were used to isolate meniscus endothelial cells for downstream analysis, making it more reliable. The scRNA-seq analysis confirmed that the frequency of meniscus endothelial cells dropped to 1% in patients with OA, and flow cytometry analysis of freshly isolated meniscus biopsies confirmed this tendency. Furthermore, this phenomenon revealed that the cells underwent degeneration and injury.

Although OA has long been considered a primary degenerative disease characterized by an injured joint, the abnormal microenvironment of the subchondral bone has attracted attention in recent years [3]. This study confirmed that the blood vessels in the meniscus of patients with OA underwent pathological variations. Based on a high-throughput genetic profile, this study initially reported that meniscus endothelial cells contain two subclusters, each of which could be identified by feature genes: HOXA13 and RASGRF2. Interestingly, HOXA13 has been reported to be critical for vascular patterning [34, 35], and RASGRF2 is involved in the response to endoplasmic reticulum stress in endothelial cells [36]. The drastic upregulation of the expression of these two genes in the meniscus endothelial cells of patients with OA indicated disordered cellular biological features, which inevitably contributed to the pathological meniscus microenvironment in patients with OA.

In addition, in patients with OA, both endothelial cell subclusters showed vigorous expression of APLNR (coding the receptor for apelin), a marker for injured and apoptotic endothelial cells [12]. Decreased endothelial cell numbers in the meniscus of patients with OA support this hypothesis. In contrast, a higher expression of APLNR could serve therapeutic purposes since its ligand, apelin, has an antiapoptotic effect [9]. Consistently, the downregulated expression of APLN has been observed in both meniscal endothelial cells in patients with OA, which could result in enhanced apoptosis of endothelial cells. Unexpectedly, two intrinsic apoptosis factors, CASP3 and BID, were upregulated in two endothelial cell subclusters in patients with OA. Downstreaming cell culturing of purified meniscus endothelial cells from patients with OA showed a pronounced outcome. This study demonstrated that apelin could function as a therapeutic agent against OA by protecting the meniscus endothelial cells.

Moreover, apelin also possesses the capability of controlling blood pressure [37], promoting angiogenesis [38], and interacting with ACE2, the main receptor for novel coronavirus COVID-19 [39, 40]. Apelin has been reported to rescue heart failure potentially and pulmonary arterial hypertension [41], two syndromes frequently reported from COVID-19 infected patients [42, 43]. Therefore, evaluating the mentioned perspectives with biopsies from COVID-19 infected patients will help develop therapeutic strategies against the COVID-19 pandemic.

## Figures and Tables

**Figure 1:** Identification of endothelial cells in meniscus biopsies. (a) scRNA-seq analysis of cellularity in meniscus: the left UMAP plot shows nine clusters across 3577 meniscus cells isolated from controls, and the right UMAP plot shows 11 clusters across 3256 meniscus cells isolated from patients with OA. (b) Violin plots showing the expression of endothelial cell feature genes (CD93, CDH5, and PECAM1) and monocyte/macrophage feature genes (CD14 and MS4A7). (c) Left pie plot showing the proportion of nine clusters in controls and the right pie plot showing the proportion of nine clusters in patients with OA. (d) Flow cytometry analysis gating on endothelial cells. Endothelial cells were gated on 7-AAD-CD45-PECAM1+ cells. 4 × 10^5^ cells were acquired from each sample. (e) Dot plot showing statistical analysis of the absolute number of meniscus endothelial cells between controls and patients with OA. Each dot represents one readout. Data represent four independent experiments. ^∗∗^*p* < 0.01.

**Figure 2:** Heterogeneity of endothelial cell in meniscus biopsies. (a) UMAP plot showing integrated analysis of meniscus endothelial cells. (b) Violin plots showing the expressions of feature genes in endothelial subclusters (HOXA13 and RASGRF2). (c) Heatmap showing the disparity of the top 10 genes between meniscus endothelial cell subclusters. (d) Gene set enrichment analysis showing meniscus endothelial cell subclusters exhibits distinguished biological features. (e) Split UMAP plots showing the comparison of meniscus endothelial cell subclusters between controls and patients with OA. (f) Flow cytometry analysis showing differences of meniscus endothelial cell subclusters between controls and patients with OA. 4 × 10^5^ cells were acquired from each sample. (g) Dot plot showing statistical analysis of the absolute number of endothelial cell subclusters between controls and patients with OA. Each dot represents one readout. Data represents three independent experiments. ^∗∗∗^*p* < 0.001.

**Figure 3:** DEGs of meniscus endothelial cell subclusters. (a) Left volcano plot shows DEGs of endothelial subcluster EC (HOXA13), and the right volcano plot shows DEGs of subcluster EC (RASGRF2). Data were calculated as OA biopsies against controls. The DEGs with log_2_ fold change > 1 and *p* value <0.05 were considered to be upregulated (red dots), and DEGS with log_2_ fold change < −1 and *p* value <0.05 were considered to be downregulated (blue dots). Genes of interest are indicated in red. (b) qPCR result showing downregulated expression of APLN in meniscus endothelial cells of patients with OA (*n* = 7) compared with the controls (*n* = 10). Data represent three similar experiments. ^∗∗^*p* < 0.01. (c) Flow cytometry analysis of surface expression of APLNR on meniscus endothelial cell subclusters. (d) Upper dot plot showing statistical analysis of surface expression of APLNR on meniscus endothelial cell subcluster EC (HOXA13), between controls and patients with OA. The lower dot plot showing statistical analysis of surface expression of APLNR on meniscus endothelial cell subcluster EC (RASGRF2), between the controls (*n* = 6) and patients with OA (*n* = 12). Each dot represents a readout. Data represent two similar experiments. ^∗∗^*p* < 0.01. (e) Violin plots showing the expression of intrinsic apoptosis gene (CASP3, BID, and CASP7) and extrinsic apoptosis genes (FAS, TNFRSF1A, and TNFSF10) in endothelial subclusters and in meniscus endothelial cells, between controls and patients with OA.

**Figure 4:** APLN alleviates apoptosis of meniscus endothelial cells isolated from OA patients by inhibiting intrinsic apoptosis genes. Meniscus endothelial cells were isolated from patients with OA and cultured in a conditioned medium. Four groups were included: the control group indicating endothelial cells cultured in conditioned medium, the second group treated with BSA, the third group treated with apelin (APLN), the fourth group was treated with apelin (APLN) and ML221 (blocking APLNR). Six wells in each group. (a) FACS charts showing apoptotic analysis of cultured meniscus endothelial cells among four groups. (b) Box blot showing statistical analysis of early apoptotic (annexin V + PI-) cells. Six wells in each group. NS: not significant; ^∗∗^*p* < 0.01; ^∗∗∗^*p* < 0.001. Data represent three independent experiments. (c) Box plots showing the expression level of CASP3 and BID in cultured endothelial cells among the above four groups. NS: not significant; ^∗^*p* < 0.05, ^∗∗∗^*p* < 0.001. Data represent two independent experiments. (d) The upper histography showing the intracellular staining of cleaved caspase 3 (CASP3) in the meniscus endothelial cell subcluster EC (HOXA13) among the four groups. The lower dot plot shows statistical analysis of mean fluorescence intensity (MFI) for cleaved caspase 3 among the four groups. Each dot represents a readout. NS: not significant; ^∗∗^*p* < 0.01, ^∗∗∗^*p* < 0.001. The data represent two independent experiments. (e) The upper histography shows the intracellular staining of cleavage site Bid in meniscus endothelial cells subcluster EC (RASGRF2) among four groups. The lower dot plot shows statistical analysis of MFI of cleavage site Bid among the four groups. Each dot represents one read. NS: not significant. ^∗^*p* < 0.05, ^∗∗^*p* < 0.01. Data represent two independent experiments.

## Data Availability

The data and code generated or analyzed in this study are available from the corresponding author upon reasonable request.

## Abbreviations

OA: Osteoarthritis
HOXA13: Homeobox A13
RASGRF2: Ras protein-specific guanine nucleotide releasing factor 2
CASP3: Caspase 3
BID: BH3-interacting domain death agonist
APLN: APJ endogenous ligand.

## Supplementary Materials

Supplementary 1 Supplementary Figure 1: the purity of isolated meniscus endothelial cells. (a) Comparison of the endothelial cell purity before and after sorting, tested by flow cytometry. Endothelial cells were labeled with anti-PECAM1. (b) Immunofluorescent imaging of sorted endothelial cells. Endothelial cells were labeled with anti-PECAM1 (red), and nuclei were labeled with DAPI (blue).

Supplementary 2 Supplementary Figure 2: feature plots showing expression of endothelial cell feature genes (CD93, CDH5, and PECAM1) and monocyte/macrophage feature genes (CD14 and MS4A7).

Supplementary 3 Supplementary Figure 3: violin plots showing the expressions of APLN and APLNR in meniscus endothelial cell subclusters.

Supplementary 4 Supplementary Table 1: integrated EC DEGs.

Supplementary 5 Supplementary Table 2: DEGs of EC (HOXA13).

Supplementary 6 Supplementary Table 3: DEGs of EC (RASGRF2).
